# The Effects of Probiotics Supplementation on Clinical Status and Biomarkers of Oxidative Damage and Inflammation in Children with Brucellosis: A Randomized, Double-Blind, and Placebo-Controlled Trial

**DOI:** 10.1155/2022/2541117

**Published:** 2022-08-22

**Authors:** Noushin Zamani, Zeinab Ganjy, Mohammad Reza Sharif, Abbas Taghavi Ardakani, Davood Kheirkhah, Mansour Sayyah, Ali Azimi, Alireza Sharif

**Affiliations:** ^1^Infectious Diseases Research Center, Kashan University of Medical Sciences, Kashan, Iran; ^2^Clinical Research Development Unit, Shahid Beheshti Hospital, Kashan University of Medical Sciences, Kashan, Iran; ^3^Department of Pediatrics, Faculty of Medicine, Kashan University of Medical Sciences, Kashan, Iran

## Abstract

**Background:**

Increased levels of inflammatory cytokines and oxidative damage may play crucial roles in the pathogenesis of brucellosis. The purpose of this trial was to evaluate the impact of probiotics administration on clinical status and biomarkers of oxidative damage and inflammation in pediatric patients diagnosed with brucellosis.

**Methods:**

This randomized, double-blind, and placebo-controlled trial was performed by recruiting 40 patients, 8–15 years of age, who had been diagnosed with brucellosis. Study participants were randomly allocated into two groups to receive either probiotics supplement or placebo (*n* = 20 each group) for 8 weeks. Blood samples were collected at the onset and after 8 weeks of intervention to quantify biochemical parameters. Clinical status was examined by a pediatric infectious disease specialist.

**Results:**

Following 8-week intervention, probiotics supplementation substantially improved total antioxidant capacity (*P* < 0.001) and malondialdehyde (*P*=0.002). Furthermore, the difference between probiotics group and placebo group for the duration of fever (*P*=0.02) and musculoskeletal pain (*P*=0.001) was statistically significant, though probiotics administration had no significant effects on high-sensitivity C-reactive protein, total glutathione, and other clinical outcomes compared with placebo.

**Conclusion:**

Overall, probiotics intake had beneficial impact on clinical status and body antioxidative defense system in pediatric patients with brucellosis.

## 1. Introduction

Brucellosis is a zoonotic disease which is extensively distributed in rural Mediterranean regions [1]. In addition to health concerns in humans, the disease can result in serious problems in livestock, including reduced milk production, abortion, sterility, and infertility, all of which have significant implications for public health and economics [2]. Increased levels of inflammatory cytokines and oxidative damage may play crucial roles in the pathogenesis of brucellosis [3]. Oxidative damage is defined as an overproduction of reactive oxygen species (ROS) or an insufficient amount of ROS cleavage that can cause the development of lipid peroxidation, DNA damage, enzyme deactivation, and cell necrosis and apoptosis [4].

Probiotics, which are known as the living microorganisms, have been identified to have important health benefits if adequately consumed [5, 6]. Probiotics can be of clinical utilization in chronic conditions such as autoimmune disorders, gastrointestinal illness, nonalcoholic fatty liver disease, and diabetes mellitus [7–9]. Several studies in rat models and humans have documented the beneficial impact of probiotics supplementation on the levels of oxidative damage biomarkers and inflammation [10, 11]. Zanganeh et al. [3] indicated that brucellosis enhances oxidative damage biomarkers in patients. Probiotics have been demonstrated to act as a protector against oxidative damage by decreasing the pH of the intestine, producing antibacterial agents including diacetyl, hydrogen peroxide, lactoperoxidase, and acetaldehyde, removal of bacterial infections, production of some digestive enzymes and vitamins, elimination of carcinogens which causes a decrease in levels of inflammatory cytokines and hydroxyl and superoxide radicals, and the increase of glutathione peroxidase [12, 13]. Furthermore, recent meta-analyses showed probiotics supplementation can considerably improve inflammatory status and oxidative stress biomarkers in humans [14–16].

Considering the antioxidant and anti-inflammatory properties of probiotics in humans, it seems to be necessary to investigate the impact of probiotics administration in children with brucellosis. Accordingly, in this trial, we made an attempt to evaluate the effects of probiotics supplementation on clinical status and biomarkers of oxidative damage and inflammation in pediatric patients with brucellosis.

## 2. Materials and Methods

The present randomized clinical trial has been registered in the Iranian website for registration of clinical trials with the special ID of IRCT20170513033941N65 (https://www.irct.ir/trial/42614) after approval by the research ethics committee of Kashan University of Medical Sciences (KAUMS) and followed the Declaration of Helsinki and Good Clinical Practice guidelines. Current investigation included 40 pediatric patients aged 8–15 years old, had been diagnosed with brucellosis, and referred to the pediatric infectious diseases clinic of Shahid Beheshti Hospital (Kashan, Iran) affiliated to KAUMS between September 3, 2019, and February 17, 2022. The brucellosis diagnosis was on the basis of clinical manifestations and serologic tests. Patients with immunosuppressive disease and children who are receiving any immunosuppressive drugs and taking any antioxidant or anti-inflammatory agents within 12 weeks before intervention were not included. Participants were randomly allocated into two intervention groups. A randomization list was created from 1 to 40 by a random number generator website and children were randomly assigned into two groups to receive either probiotics or placebos. The block randomization method with 1 : 1 ratio was applied. The medical team, parents, children, and data assessors were blinded to treatment allocation. All participants' parents were informed about the protocol of this trial and its purposes, and the written informed consent was taken.

### 2.1. Intervention

According to our guidelines for the management of brucellosis, at admission time, all patients were treated by antibiotics (doxycyclin and rifampin). One group received probiotics capsules (Zisttakhmir Co., Tehran, Iran) including *Lactobacillus acidophilus, Bifidobacterium bifidum*, *Lactobacillus reuteri*, and *Lactobacillus fermentum* (2 × 10^9^ CFU/g each) daily for 8 weeks orally and another group received matched placebo capsules (Zisttakhmir Co., Tehran, Iran) as soon as possible after randomized allocation. All children received standard treatment of brucellosis.

### 2.2. Outcome Measures

Primary outcome was considered serum C-reactive protein (CRP) levels, but clinical status and biomarkers of oxidative damage were considered as the secondary outcomes. The two intervention groups were clinically examined by a pediatric infectious disease specialist (MS) and followed based on symptoms including chills, fever, sweating, musculoskeletal pain, and anorexia. CRP values were measured by ELISA kit (LDN, Germany), total antioxidant capacity (TAC) utilizing the method described by Strain and Benzie [17], total glutathione (GSH) by Beutler et al. method [18], and malondialdehyde (MDA) values were quantified by the spectrophotometric analysis [19].

### 2.3. Sample Size Calculation

We utilized a clinical trial sample size calculation formula where type one and type two errors were 0.05 and 0.20, respectively. The sample size was determined according to a report by Sanaie et al. [20] to compare the impact of placebo and probiotics on serum CRP levels. Using the formula, we needed 15 subjects in each group; after allowing for 35% dropouts, the final sample size was 20 subjects in each group.

### 2.4. Statistical Analyses

The normality of data was determined by the Kolmogorov–Smirnov test. To find out significant changes in continuous variables between the two groups, we applied the independent *t*-tests. The Fisher's exact and Pearson chi-square tests were utilized to compare categorical variables. Analysis of covariance was used to evaluate the impact of probiotics administration on study outcomes after adjusting for confounding parameters including age and baseline values. *P* value less than 0.05 was considered as statistically significant. All analyses were performed by the use of SPSS software version 16 (Chicago, Illinois, USA).

## 3. Results

As revealed in this study flow diagram (Figure 1), we enrolled 40 pediatric patients with brucellosis in this study; however, 3 participants were excluded from the trial because of personal reasons. Finally, 37 participants (placebo (*n* = 18) and probiotics (*n* = 19)) completed the trial. No side effects were reported following the intake of probiotics and placebo in pediatric patients with brucellosis throughout the trial.

Baseline characteristics of participants were not statistically different between the two groups (Table 1).

The difference between the probiotics group and the placebo group for the duration of fever (*P*=0.02) and musculoskeletal pain (*P*=0.001) was statistically significant; other clinical parameters did not reveal any significant difference (Table 2).

Following 8-week intervention, probiotics supplementation substantially improved TAC (*P* < 0.001) and MDA (*P*=0.002), though probiotics had no considerable impact on hs-CRP and GSH compared with placebo (Table 3).

## 4. Discussion

To our best knowledge, present trial was the first investigation to report on the favorable impact of 8 weeks of probiotics consumption on clinical status and biochemical parameters in children with brucellosis. We uncovered that probiotics administration decreased the duration of musculoskeletal pain and fever, and plasma MDA and substantially increased total antioxidant capacity. Supplementation with probiotics in children with brucellosis had no significant impact on the other outcomes.

Brucella species are facultative intracellular bacteria that cause chronic infection in humans [21]. Previous studies have shown that infectious diseases activate various immune cells that produce free oxygen radicals, which lead to the killing of intracellular and extracellular microbes [22]. The free radicals are vital molecules that kill bacteria inside phagocytes through peroxidation of fatty acids, proteins, and DNA [23]. However, overproduction of free radicals can lead to cell apoptosis via impaired DNA replication and damage to DNA polymerase [24].

Probiotics may benefit pediatric patients with brucellosis through its promising effects on biomarkers of oxidative stress and inflammatory status [14, 21]. Several interventional studies have investigated the impact of probiotics intake on inflammatory cytokines and antioxidative defense systems, but the findings have been inconsistent. In a study conducted by Villar-García et al. [25], probiotics administration to people with HIV for 12 weeks significantly reduced serum levels of inflammatory mediators such as IL-6 and hs-CRP. Consumption of probiotics supplements containing *Lactobacillus acidophilus, Lactobacillus rhamnosus*, and *Bifidobacterium bifidum* for 8 weeks by individuals with inflammatory bowel syndrome resulted in considerable decrement in serum CRP levels [26]. Raygan et al. [10] documented that probiotics intake containing *Bifidobacterium bifidum*, *Lactobacillus acidophilus*, and *Lactobacillus casei* (2 × 10^9^ CFU/g each) substantially reduced hs-CRP and increased serum levels of TAC and GSH in diabetic people with coronary heart disease, but did not influence other antioxidant markers. Furthermore, three months administration of multispecies probiotics supplements to hemodialysis patients ameliorated antioxidant defense system and inflammatory status [27]. However, probiotics supplementation (*Lactobacillus salivarius*) for 6 weeks in overweight adolescents did not affect inflammatory cytokines including serum CRP, IL-6, and TNF-alpha concentrations [28]. Moreover, Sherf-Dagan et al. [29] revealed that intake of probiotics for one month did not influence oxidative damage biomarkers and inflammatory status. The anti-inflammatory and antioxidative impact of probiotics may be due to decreasing production of hydrogen peroxide radicals [30], inhibiting of nuclear factor-*κ*B [31], and producing short-chain fatty acids in the gut [32, 33].

Prior studies have indicated the beneficial effects of short-term or long term probiotics supplementation in the treatment of infectious and inflammatory diseases. Najafi et al. [34] revealed that probiotics administration (for 5 days) to people with bacterial pneumonia considerably reduced the mean duration of cough, hospitalization, tachypnea, dyspnea, and fever. Corsello et al. [35] documented that probiotics consumption (*Lactobacillus paracasei*) is an efficient strategy in preventing common infectious diseases such as gastroenteritis, pharyngitis, laryngitis, and tracheitis in children. Furthermore, Cardenas et al. [36] demonstrated administration of probiotics (1 × 10⁸ CFU of *Lactobacillus salivarius* daily for 6 months) can lead to a significant decrease in the number of acute otitis media episodes during the study period. Additionally, Shida et al. [37] showed probiotics supplementation reduces the incidence and duration of upper respiratory tract infections in healthy middle-aged individuals by modulating the immune system and preventing natural killer cell activity in peripheral blood mononuclear cells. Finally, probiotics intake resulted in a significant reduction in risks for gastrointestinal and respiratory tract infections in children [38]. Previous investigations documented that probiotic has a safety profile without any serious side effects. Only minimal adverse effects such as transient gastrointestinal symptoms, nausea, excessive gassiness, bloating, and diarrhea have been reported [39].

The limitations to this trial include small sample size, the short period of intervention, and lack of examinations for fecal bacteria load before and after probiotics intake. Also, due to inappropriate funding, there was no chance to evaluate other biomarkers of oxidative damage and inflammatory mediators as well as gene expression related to inflammation and oxidative stress in pediatric patients with brucellosis. Our study has no enough power to analyze data for stratified results due to small sample size. Also, the number of females was low; therefore, we could not analyze data based on gender. Future studies with a larger sample size, longer period of intervention, and various species of probiotics might aid in a better understanding of the favorable impact of probiotics supplementation in children with brucellosis.

## 5. Conclusions

Overall, probiotics consumption for 8 weeks had promising effects on body antioxidative defense system and clinical status such as duration of musculoskeletal and fever in pediatric patients with brucellosis. Our findings clarify that probiotics administration as adjunctive therapy along with antibiotic therapies may have favorable therapeutic impact.

## Figures and Tables

**Figure 1:** Summary of patient flow diagram.

**Table 1:** General characteristics of study participants.

	Placebo group (*n* = 18)	Probiotics group (*n* = 19)	*P* ^1^
Age (y)	11.3 ± 2.2	10.7 ± 2.3	0.41†

Gender			0.64
Male	10 (55.6)	12 (63.2)	
Female	8 (44.4)	7 (36.8)	

Place of residence			0.82
Urban	6 (33.3)	7 (36.8)	
Rural	12 (66.7)	12 (63.2)	

Nationality			0.92
Iranian	13 (72.2)	14 (73.7)	
Non-Iranian	5 (27.8)	5 (26.3)	

Data are presented as mean ± SD or numbers (%). ^1^Obtained from chi-square test. †Obtained from independent *t*-test.

**Table 2:** Clinical status of pediatric patients with brucellosis.

Symptom duration (day)	Placebo (*n* = 18)	Probiotics (*n* = 19)	*P* ^*a*^
Fever	6.4 ± 2.5	4.7 ± 1.9	**0.02**
Chills	5.5 ± 2.2	4.3 ± 1.8	0.09
Musculoskeletal pain	16.5 ± 3.9	12.3 ± 2.9	**0.001**
Anorexia	12.1 ± 2.3	11.2 ± 1.4	0.18
Sweating	8.3 ± 2.1	7.5 ± 1.6	0.17

Data are presented as mean ± SD. ^a^Obtained from independent *t*-test.

**Table 3:** Biochemical parameters at baseline and after the 8-week intervention in children with brucellosis that received either probiotics or placebo.

Variables	Placebo group (*n* = 18)		Probiotics group (*n* = 19)		*P* ^1^
	Baseline	Week 8	Baseline	Week 8	
Hs-CRP (mg/L)	16.7 ± 6.8	6.5 ± 3.5	16.5 ± 6.9	5.6 ± 2.5	0.13
TAC (mmol/L)	330.1 ± 53.8	762.9 ± 69.5	324.5 ± 91.7	1043.1 ± 126.8	**<0.001**
GSH (*µ*mol/L)	664.1 ± 189.6	743.1 ± 209.6	540.5 ± 87.1	608.0 ± 84.8	0.60
MDA (*µ*mol/L)	7.7 ± 0.7	4.2 ± 0.4	7.3 ± 0.9	3.4 ± 1.0	**0.002**

^1^Obtained from ANCOVA (values are adjusted for baseline values and age). GSH, total glutathione; hs-CRP, high-sensitivity C-reactive protein; MDA, malondialdehyde; TAC, total antioxidant capacity.

## Data Availability

The primary data for this trial are available from the corresponding author on reasonable request.
